This article has been retracted.

# Analysis of the Correlation between the Level of Posttraumatic Growth and Social Support among Caregivers of Children with Acute Leukemia

**DOI:** 10.1155/2022/7456284

**Published:** 2022-09-07

**Authors:** Qiurong Chen, Xujia Xiao, Yaling Zhang, Chao Lin

**Affiliations:** ^1^Department of Pediatric Hematologic Oncology Nursing, West China Second University Hospital, Sichuan University/West China School of Nursing, Sichuan University, Chengdu 610041, Sichuan, China; ^2^Key Laboratory of Birth Defects and Related Diseases of Women and Children, Sichuan University, Ministry of Education, Chengdu 610041, Sichuan, China; ^3^West China School of Nursing, Sichuan University, Chengdu 610041, Sichuan, China; ^4^Department of Pediatric Hematologic Oncology, West China Second University Hospital, Sichuan University, Chengdu 610041, Sichuan, China

## Abstract

We investigate the current situation of stress burden and quality of life of primary caregivers of children with leukemia and analyze the correlation between their stress burden and quality of life, using the phenomenological research method in qualitative research. The posttraumatic growth experiences of the parents of children with leukemia included life perceptions (appreciation of life, change in priority of important things in life, and adjustment of self to reality); personal empowerment (increased sense of self-reliance and increased sense of self-achievement); and improvement of interpersonal relationships (increased family harmony, valuing parent-child bonding, benefiting from professional support from other parents and medical staff, and increased sense of empathy and altruism). The posttraumatic growth experiences of parents of children with leukemia are based on their roles (parenting) and responsibilities and can be used as an important basis for future trauma interventions, as well as an entry point for exploring the posttraumatic growth potential of parents of children with leukemia and ultimately improving the posttraumatic growth of parents of children with leukemia.

## 1. Introduction

According to statistics, the incidence of leukemia in children under 14 years of age is 25% [1, 2] and requires prolonged care by their relatives, especially during hospitalization, causing numerous physical and psychological problems for the child's primary caregiver, such as varying degrees of stress, anxiety, frustration, disappointment, and denial during the early stages of diagnosis, even after the child's disease is controlled [3, 4]. These problems may persist for years even after the child's disease is controlled [5, 6]. When a child is diagnosed with leukemia, the entire family may also face challenges such as unemployment, helplessness, financial distress, disrupted relationships, or inability to participate properly in social activities [7].

The stressful, emotional reactions of the primary caregiver to such problems are referred to as “caregiver reactions” [8]. The quality of life (QOL) of primary caregivers of patients with acute leukemia has long been a priority for clinical caregivers [9]. Childhood leukemia is a chronic, systemic, and recurrent disease, and parents play an important role in the long-term course of the child's illness. Previously, domestic and international studies on parents of affected children have often focused only on their negative emotions, cognition, and behavior [10].

In recent years, influenced by positive psychology research, foreign researchers have shifted from focusing only on stress, deficits, and illness to tapping into an individual's own strengths and potential, and more and more studies have found that a high-stress life event and the threat of death or illness can be a trauma or an opportunity for self-growth that renews self-perceptions and thus makes positive adjustments in psychological behavior [11, 12]. We refer to this growth as “posttraumatic growth (PTG). Posttraumatic growth is a theoretical concept born in the American cultural context, and the perception of traumatic events, the content of posttraumatic growth, and the influencing factors involved in the growth process may differ in different cultural contexts.

Acute leukemia is a global problem, and according to the International Agency for Acute Leukemia Research (IARC), 22.2 million people are expected to suffer from acute leukemia by 2030 [13]. The incidence and mortality rate of acute leukemia in China is increasing year by year, and the statistics of acute leukemia in 2017 showed that 4.29 million new cases of acute leukemia occur each year, accounting for 20% of new cases and 2.81 million deaths worldwide [14]. Acute leukemia has become a major cause of death and a major public health problem for the population in China [15]. With the continuous improvement of medical technology and improvement, the 5-year survival rate of acute leukemia patients is as high as 68%, in which the careful care of caregivers is one of the important reasons for their extended survival time. Caregivers can have a negative impact on their physical and mental health due to the heavy caregiving tasks and psychological stress [16, 17]. Related studies confirmed that the negative psychological state of caregivers decreases the quality of care, which in turn reduces the quality of life of patients with acute leukemia. Although caregivers of patients with acute leukemia face great difficulties and challenges in the process of caregiving, some of them also perceive positive meaning and make positive changes in their lives, which is called “sense of benefit from illness,” also known as benefit finding (BF), in which individuals perceive their personal experiences from negative life events such as illness or trauma. This positive change is called “illness benefit,” also known as benefit finding (BF), which is a cognitive and behavioral adaptation process in which individuals perceive personal, social, psychological, and spiritual benefits from the experience of negative life events such as illness or trauma [18, 19]. Studies have shown that the lower the sense of benefit from illness, the worse the physical and mental health. Social support is an important predictor of perceived illness benefit, and caregivers with higher social support have a higher perception of illness benefit, as well as a significantly improved quality of life for the caregiver [20]. Self-efficacy reflects the extent to which individuals realize their potential, which can be improved through learning, and higher self-efficacy indicates that acute leukemia caregivers have greater self-confidence in their ability to cope with caregiving tasks [7, 21–23]. Previous studies have focused on correlations between variables, but fewer studies have examined how self-efficacy plays a role in the relationship between social support and perceived benefit from illness among caregivers of hospitalized acute leukemia patients. In this paper, using a phenomenological approach in qualitative research, 286 caregivers of hospitalized acute leukemia patients were selected as the study population, and a one-on-one interview was conducted using a semi-structured interview outline guided by selecting one of the parents of the affected children to participate in the interview [24]. The aim of this study was to investigate the intrinsic link between self-efficacy, social support, and sense of illness benefit among caregivers of hospitalized acute leukemia patients, and to clarify their mediating effects, with the aim of improving caregivers' self-efficacy by increasing their social support, thus providing a theoretical basis for enhancing their sense of illness benefit [25].

## 2. Materials and Methods

### 2.1. General Information

A convenience sampling method was used to select 286 caregivers of hospitalized acute leukemia patients in our hospital as the study population. Inclusion criteria for caregivers are as follows: ① patients with pathologically diagnosed acute leukemia; ② caregivers aged ≥18 years; ③ patients' primary caregiver, who could be the patient's spouse, children, or other relatives, to undertake the primary caregiving tasks; ④ patients with unpaid care; ⑤ patients with ability to read and understand text; and ⑥ patients with informed consent and cooperation with the survey. Exclusion criteria are as follows: significant negative life events in the last 3 months and mental or intellectual disability.

A purposive sample of 10 fathers or mothers of children with leukemia who attended the pediatric department of Peking Union Medical College Hospital from May 2015 to February 2016 was selected for the interview. Inclusion criteria are as follows: (i) the child's disease met the diagnostic criteria for leukemia; (ii) they assumed the primary responsibility for caring for the child (at least 6 hours per day); and (iii) they were willing and able to fully express their true experiences and feelings. The sample size was based on data saturation.

### 2.2. Research Methodology

A semi-structured interview was used to collect data, guided by the phenomenological approach in qualitative research. In this paper, a one-on-one interview was used, in which one of the parents of the affected child was selected to participate in the interview, and the number of interviewees was determined to reach data saturation. Each interviewee was referred to as a case in the study, and interviewers were numbered in order from A–J. The researcher used a semi-structured interview outline as a guide to conduct the interviews. ① How did you feel when your child's illness was first diagnosed? ② What changes did you experience during the course of your child's illness? ③ Did you have any positive/positive changes during the course of your child's illness? ④ What factors led you to make these positive changes? Use the above questions to ask parents of children with leukemia about their posttraumatic growth experiences.

### 2.3. Data Collection and Analysis Methods

The researcher indicated the purpose of the study to the study participants, signed an informed consent form, and agreed on the time and place of the interview. Each interview was recorded for 30–45 minutes. The researcher listened carefully and recorded the interview contents and the expressions and emotional changes of the interviewees. After the interviews were completed, the audio recordings were transcribed into text and analyzed using Colaizzi's analysis [12], and meaningful statements that were consistent with the posttraumatic growth experience of the parents of the children with leukemia were extracted, summarized, refined, and further formed into themes and thematic clusters for a complete narrative. Finally, the results obtained were returned to the interviewees to further verify the authenticity of the content.

## 3. Research Tools

The Chinese version of the Benefits of Caregiver Illness Scale (BFS-C) is used to understand the level of benefits of caregiver illness. The Chinese version of the scale has 17 items, including three dimensions of personal growth (items 9–17), interpersonal improvement (items 4–8), and acceptance (items 1–3). The scale uses the 5-point Likert scale, with scores of 1–5 representing “not at all,” “a little,” “moderately,” “a lot,” and “very much,” respectively. The higher the score, the higher the level of the caregiver's sense of benefit from illness. Cronbach's *α* coefficient of the Chinese version of the Sense of Benefit Scale is ≥0.819, with good reliability and validity.

### 3.1. Social Support Rating Scale

The total social support score, which is 66 out of 66. A total score of ≤22 is considered low, 23–44 is medium, and 45–66 is high. The retest reliability of the scale is 0.89–0.94, which is applicable to Chinese population.

### 3.2. General Self-Efficacy Scale (GSES)

The GSES was first developed by Schwarzer, a German professor of psychology, together with his colleagues, and the scale has been translated into several languages and is widely used internationally. The Chinese version of the GSES, which was translated and revised in 2001, is a unidimensional scale with 10 items, and each item is rated on a 4-point Likert scale, with scores from 1 to 4 representing “not at all correct,” “fairly correct,” “mostly correct,” and “completely correct,” respectively. The lower the score, the lower the level of general self-efficacy. A score of <20 indicates a low level of general self-efficacy; a score of 20–30 indicates a medium level; and a score of >30 indicates a high level. After measurement, Cronbach's *α* was 0.87, and the scale had good reliability.

## 4. Results

### 4.1. Scores of Perceived Disease Benefit, Social Support, and Self-Efficacy of Caregivers of Hospitalized Acute Leukemia Patients

Caregivers of hospitalized patients with acute leukemia had a total score of (66.70 ± 10.8) for perceived benefit of illness, with scores for each dimension being personal growth (35.2 ± 6.7), interpersonal relationship (21.2 ± 3.4), and acceptance dimension (10.6 ± 2.7); the highest mean score for the interpersonal relationship dimension was (4.23 ± 0.68); the lowest mean score for the acceptance dimension was (2.11 ± 0.54). The total score of social support for caregivers of hospitalized acute leukemia patients was (42.6 ± 6.8), and the scores of each dimension were (9.7 ± 3.4) for objective support, (25.9 ± 4.2) for subjective support, and (7.02 ± 1.83) for utilization of support; among them, the mean score of the subjective support dimension entry was the highest (6.48 ± 1.04); the mean score of the utilization of support dimension entry was the lowest (2.11 ± 0.54). The lowest mean score was (2.33 ± 0.61). The total score of self-efficacy of caregivers of hospitalized acute leukemia patients was (26.1 ± 6.41).

### 4.2. Correlation Analysis of Caregivers' Perceptions of Disease Benefit, Social Support, and Self-Efficacy in Hospitalized Acute Leukemia Patients

The results of this study showed that the total illness benefit score and self-efficacy was positively correlated with illness benefit, personal growth, interpersonal relationships, and acceptance, as shown in Table 1.

### 4.3. Self-Efficacy between Social Support and Perception of Illness Benefit

The regression analysis showed that all four standardized regression coefficients reached a significant level (*P* < 0.01), and the mediating effect of self-efficacy between social support and perception of illness benefit is shown in Table 2 and Figure 1.

### 4.4. Change in Priority of Important Things in Life

Prior to the child's illness, parents often have high expectations and goals for themselves and for their child's life, and the child's illness causes the hopes to be dashed. After a period of self-adjustment, parents change their previous ranking of priorities in life and become more aware of what is most important in life. Most parents believe that being healthy and having a happy life is the most important thing. For example, Mother D said “Besides life and death, everything else is trivial; to be alive, to be healthy and safe is the most important thing.” Father E said “In the past, when the child did not have the disease, I always thought of working hard to save some money for the child in the future, but later, when the child got sick, I did not want to think so much, it does not matter how high or low the income is, the family is healthy and happy life is the most important.” In the face of the high cost of medical care for their children, some parents say that money is the most important thing. For example, Father F said “In the past, the focus of life was food, clothing, housing and transportation, but now I think money is the most important thing, do everything to save up for the child's next treatment, as long as there is money, to come to the child's medical care” (Table 3).

### 4.5. Adjustment of Self-Acceptance of Reality

Stress burden and quality of life scores of primary caregivers of children with leukemia. Caregiver quality of life scores (13.9 ± 3.2) and total stress burden scores averaged (72.6 ± 11.7), as shown in Table 4.

Pearson correlation analysis of stress burden and quality of life of primary caregivers of children with leukemia (Table 5).

### 4.6. Personal Empowerment

During the interview, some parents (B, D, H, and I) expressed their reluctance to let neighbors and friends know about their children's illness and their reluctance to communicate with others, trying to alleviate their suffering by being alone. The distance from social resources directly led to a decrease in the level of social support and an increased sense of self-reliance. For example, Mother I said “I don't talk to my family now (about my child's illness) because I don't want them to worry, and I talk to my colleagues too.”

Mother B said “I don't want everyone to know that my child is sick, I just know how to solve the problem myself.” In addition, a few parents of children with the disease said that they received more social support at the beginning of the disease, but in the long run, social support is difficult to sustain, such as Father F said “When the child first got sick, there were many friends who cared, but the disease cannot be cured for a while, or at all, so who can visit you every day, so to continue to live, you still have to count on yourself.”

As caregivers, the parents of the child should not only take care of the child's life, but also care about the child's mental and psychological state and good psychological guidance. In addition, they have to learn about the disease, home care, and medication, so that they can feel needed and have a greater sense of self-fulfillment in the process of caring for their children. For example, Mother B said “After the disease, my child has been out of school, so I have to tutor her homework and take up the task of educating her, and I am the child's teacher at home.” Father F: “My child has a strong competitive mind, and since he got sick, he eats less and doesn't talk much. I as a parent is mainly to guide him, psychologically comfort him, let him not anxious, relaxed mind.” Mother E: “The child is quite afraid that her classmates know she has a disease, usually she will hide it from them, and every time she comes to the hospital, she will also lie, in order to avoid the child living in a lie, I need to help the child face bravely, I also have to be responsible for the child's psychological work, cannot be well after the psychological problems.”

## 5. Discussion

### 5.1. Current Analysis of the Level of Disease Benefit Perception among Caregivers of Hospitalized Acute Leukemia Patients

The perception of disease benefit among caregivers of hospitalized acute leukemia patients was moderate. The results of this study showed that the total mean score of perception of disease benefit among caregivers of hospitalized acute leukemia patients was (66.70 ± 10.8), indicating a moderate level of perception of disease benefit among caregivers of hospitalized acute leukemia patients. Although caregivers of hospitalized acute leukemia patients experience negative effects such as financial burden and anxiety and depression during the process of caregiving, caregivers also perceive a sense of illness benefit and growth, such as learning to accept reality, appreciate the meaning of life, cherish the present moment, and have confidence and hope, increased ability to actively learn and caregiving, perceived multiple support from family, friends, and healthcare providers, and health-related cognitive behaviors. The perception of health-related cognitive behaviors improves [13]. Among the three dimensions of the BFS-C scale, the highest score for the personal growth dimension may be related to the following two factors The highest scores on the personal growth dimension of the BFS-C scale may be related to the fact that caregivers are able to self-regulate their negative emotions and have improved self-control; the overall psychological and spiritual growth of the caregiver as the caregiving time increases, as well as the acquisition of knowledge about the disease and caregiving skills.

### 5.2. Correlation Analysis of Caregiver's Social Support, Self-Efficacy, and Perception of Disease Benefit in Hospitalized Acute Leukemia Patients

The results of this study showed that social support and subjective and objective support dimensions were positively correlated with the perception of illness benefit, i.e., the higher the social support, the higher the caregiver's perception of illness benefit, which is consistent with domestic and international studies [14]. Social support is a multidimensional interaction established through formal and informal interactions with other people or organizations to obtain moral comfort, financial support, and information support [15].

Social support can provide caregivers with knowledge of disease treatment, effective caregiving skills, financial and material assistance, and spiritual support, which can help to reduce the psychological and financial burdens of helplessness, despair, and depression of caregiving patients, so that they can cope with caregiving tasks in a positive frame of mind, increase their confidence in caregiving, and easily perceive positive changes. Therefore, healthcare workers understand and pay attention to the caregiver's social support during their interactions with the caregiver and guide them to tap into more positive perceptions by increasing their social support and reducing the perception of negative emotions.

### 5.3. The Mediating Role of Self-Efficacy between Caregiver's Social Support and Perception of Disease Benefit in Patients with Acute Leukemia

The analysis of the mediating effect showed that self-efficacy partially mediated the effect between social support and perception of benefit from illness, with the mediating effect accounting for 35.53% of the total effect, indicating that social support can affect perception of benefit from illness both directly and indirectly through the mediating effect of self-efficacy, which is similar to the results of a related study in China [15]. Self-efficacy reflects the degree to which an individual realizes his or her potential, which can be improved through learning, and higher self-efficacy indicates that acute leukemia caregivers are more confident in their ability to cope with caregiving tasks [16]. When caregivers face frustration and poor mood, the higher their perceived social support, the more they will make full use of the various resources provided by healthcare professionals, family members, and friends, so that their internal self-efficacy will increase, they will take the initiative to learn about disease treatment, master caregiving skills, improve their caregiving adaptability, reduce anxiety and depression, and other negative emotions, and, at the same time, enhance the positive experience brought about by caregiving. Therefore, while providing a level of social support, clinical healthcare workers can also mobilize their own potential coping and problem-solving skills, enhance their self-confidence, and improve their sense of self-efficacy, thus producing positive changes and experiencing a greater sense of benefit from the disease and providing good care for patients.

Caregivers of hospitalized acute leukemia patients have moderate levels of illness benefit perceptions, and social support and self-efficacy are positively related to illness benefit perceptions, with social support influencing illness benefit perceptions through the mediating role of self-efficacy. Healthcare professionals can take effective interventions to improve caregivers' perceptions of illness benefit, starting from both social support and self-efficacy. In this study, only one tertiary care hospital was selected for the survey, and the sample was not representative enough. In addition, this study only examined the relationship between social support, self-efficacy, and sense of illness benefit and did not delve into the effects of the variables on the sense of illness benefit. Therefore, subsequent studies can expand the sample size and increase the variables to explore the path analysis and mechanism of action among the variables.

## Figures and Tables

**Figure 1:** Model of the mediating effect of self-efficacy between caregiver social support and perception of disease benefit in patients with acute leukemia.

**Table 1:** Correlation analysis of caregivers' sense of illness benefit, social support, and self-efficacy in hospitalized acute leukemia patients.

Project	Social support	Subjective support	Objective support	Utilization of support	Self-efficacy disorder	Disease benefit	Personal growth	Interpersonal relationship
Social support	1.00	—	—	—	—	—	—	—
Subjective support	0.83	1.00	—	—	—	—	—	—
Objective support	0.78	0.30	1.00	—	—	—	—	—
Utilization of support	0.48	0.23	0.14	1.00	—	—	—	—
Self-efficacy disorder	0.32	0.25	0.31	0.03	1.00	—	—	—
Disease benefit	0.21	0.19	0.18	0.12	0.17	1.00	—	—
Personal growth	0.23	0.22	0.18	0.02	0.30	1.00	1.00	—
Interpersonal relationship	0.04	−0.08	0.12	0.07	0.13	0.60	0.38	0.37

**Table 2:** Self-efficacy between social support and perceived benefit from illness.

Step	Independent variable	Dependent variable	*β*	S.E	*t*	*P*	*R * ^2^	*F*	*P*
Step 1	Social support	Disease benefit	0.212	0.091	3.632	<0.001	0.045	13.20	<0.001
Step 2	Social support	Self-efficacy	0.320	1.157	5.678	<0.001	0.103	32.192	<0.001
Step 3	Social support	Disease benefit	0.234	0.036	3.924	<0.001	0.095	14.667	<0.001

**Table 3:** Demographic characteristics of the interviewees (*n* = 10).

Participant	Parental role	Age (y)	Educational level	Occupation	Marital status	Gender	Age (y)	Course of disease (months)	Disease diagnosis
A	Mother	33	Undergraduate	Liberal professions	Married	Male	6	16	Juvenile idiopathic arthritis

B	Mother	45	Undergraduate	Accounting	Married	Female	12	21	Systemic lupus erythematosus

C	Father	40	High school	Individual	Married	Female	13	17	Systemic lupus erythematosus

D	Mother	41	Junior high school	Farmer	Married	Female	12	17	Takayasu arteritis

E	Mother	45	Master	Teacher	Married	Male	15	132	Systemic lupus erythematosus

F	Father	46	High school	Farmer	Married	Female	17	54	Juvenile idiopathic arthritis

**Table 4:** Caregiver stress burden and quality of life scores (points, $\bar{x}\pm s$).

Dimension	Number of entries	Highest score	Lowest score	Average score
Total score of stress burden	20	104	38	72.3±15.9
Health and time burden	8	33	15	22.6±4.0
Financial burden	3	20	8	15.0±4.3
Lack of family support	6	18	5	11.6±3.7
Self-esteem	7	43	10	23.5±4.0
Quality of life	25	113	35	79.7±13.7
Physiological field	4	18	6	14.1±3.0
Psychological field	4	20	5	12.5±3.2
Independence	4	21	8	14.9±2.0
Social relations	4	19	5	13.0±2.6
Spirit	4	15	6	10.5±2.6
Environmental field	4	20	7	14.7±2.3

**Table 5:** Pearson correlation analysis of stress burden and quality of life of primary caregivers of children with leukemia (*r*).

Dimension	Total score of stress burden	Health and time burden	Financial burden	Lack of family support	Self-esteem
Quality of life	−0.57	−0.53	−0.68	−0.58	0.54
Physiological field	−0.48	−0.50	−0.02	−0.14	0.15
Psychological field	−0.69	−0.52	−0.55	−0.63	0.15
Independence	−0.45	−0.64	−0.14	−0.69	0.06
Social relations	−0.84	−0.72	−0.48	−0.55	−0.64
Environmental field	−0.48	−0.62	−0.11	−0.06	0.21
Spiritual field	−0.10	−0.54	−0.10	−0.14	0.15

## Data Availability

Data sharing is not applicable to this article as no datasets were generated or analyzed during the current study.
